# Magnetic Resonance Imaging Images under Deep Learning in the Identification of Tuberculosis and Pneumonia

**DOI:** 10.1155/2021/6772624

**Published:** 2021-12-15

**Authors:** Yabin Liu, Yimin Wang, Ya Shu, Jing Zhu

**Affiliations:** Clinical Medical College and The First Affiliated Hospital of Chengdu Medical College, Chengdu, Sichuan 610500, China

## Abstract

This work aimed to explore the application value of deep learning-based magnetic resonance imaging (MRI) images in the identification of tuberculosis and pneumonia, in order to provide a certain reference basis for clinical identification. In this study, 30 pulmonary tuberculosis patients and 27 pneumonia patients who were hospitalized were selected as the research objects, and they were divided into a pulmonary tuberculosis group and a pneumonia group. MRI examination based on noise reduction algorithms was used to observe and compare the signal-to-noise ratio (SNR) and carrier-to-noise ratio (CNR) of the images. In addition, the apparent diffusion coefficient (ADC) value for the diagnosis efficiency of lung parenchymal lesions was analyzed, and the best *b* value was selected. The results showed that the MRI image after denoising by the deep convolutional neural network (DCNN) algorithm was clearer, the edges of the lung tissue were regular, the inflammation signal was higher, and the SNR and CNR were better than before, which were 119.79 versus 83.43 and 12.59 versus 7.21, respectively. The accuracy of MRI based on a deep learning algorithm in the diagnosis of pulmonary tuberculosis and pneumonia was significantly improved (96.67% vs. 70%, 100% vs. 62.96%) (*P* < 0.05). With the increase in *b* value, the CNR and SNR of MRI images all showed a downward trend (*P* < 0.05). Therefore, it was found that the shadow of tuberculosis lesions under a specific sequence was higher than that of pneumonia in the process of identifying tuberculosis and pneumonia, which reflected the importance of deep learning MRI images in the differential diagnosis of tuberculosis and pneumonia, thereby providing reference basis for clinical follow-up diagnosis and treatment.

## 1. Introduction

Pulmonary tuberculosis is a chronic infectious disease caused by conjugated mycobacteria. After illness, patients may experience low-grade fever (it becomes worse in the afternoon), night sweats, fatigue, anorexia, weight loss, female menstrual disorders, and other adverse reactions. Besides, there are cough, sputum expectoration, hemoptysis, chest pain of different degrees of chest tightness, or dyspnea in the respiratory tract. It varies according to the degree of the disease and the range of the lesion. In the early stage of tuberculosis, it is difficult to find positive signs in a small range, and the percussion of patients with a wide range of lesions is presented with dullness, enhanced speech fibrillation, low alveolar breathing sounds, and wet rales [1]. Advanced tuberculosis develops fibrosis, and local contraction causes pleural collapse and mediastinal displacement [1]. In patients with tuberculous pleurisy, there are pleural frictional sounds in the early stage. The chest wall is full, percussion is turbidity and solid, and speech tremors and breathing sounds decrease or disappear when a large amount of pleural effusion is formed [2]. Some patients may not develop the disease after being infected with tuberculosis. When the resistance is reduced or the cell-mediated allergy is increased, it may cause clinical disease. If timely diagnosis and reasonable treatment are given, most of them can be clinically cured, so improving diagnostic techniques is the premise of effective treatment of tuberculosis [3].

Pneumonia is mostly caused by lung infection with bacteria and viruses. The early symptoms of patients are mainly cough, fever, and shortness of breath. At the same time, they may be accompanied by symptoms such as fatigue, lethargy, dehydration, and loss of appetite [4]. For fever, the degree of fever caused by different pathogens is also inconsistent [5]. Patients with severe pneumonia symptoms may also have symptoms such as chest pain and chest tightness, which are similar to the clinical manifestations of tuberculosis. When the clinical symptoms of the two are very similar, they are not easy to be distinguished. Therefore, imaging examination methods have become the main means of identification. The imaging methods commonly used in clinical examination of lung diseases mainly include chest X-ray and CT plain film examination. However, it is found that chest X-ray films are easily affected by breathing during the detection process in clinical practice, and the measurement error is large. What is more, the radiation of computed tomography (CT) examination is large, which has a large impact on the patient, and it is not suitable for pregnant women, adolescents, and children, so its application is restricted [6]. In recent years, with the continuous development of magnetic resonance imaging (MRI) technology, the examination sequence has gradually increased. Its application in the examination of lung diseases has also risen. Due to its nonionizing radiation, multiparameter imaging, and higher soft tissue resolution, the unique advantages have gradually increased its application in pregnant women, adolescents, and children. During the examination, there are large differences in individual structures between patients, and the changes in lung tissue with respiratory work can often affect the imaging results of the image. Therefore, it is necessary to use the convolutional neural network (CNN) algorithm in in-depth learning for preprocessing to reduce the influence of other factors on the research results [7]. Many studies have proposed that deep learning algorithms have good effects on the denoising of medical images, including CNN algorithms and deep CNN (DCNN) [8–10]. Of course, good research results have been achieved in the processing of MRI images [11, 12].

Therefore, this study used MRI images based on the DCNN denoising algorithm to examine and analyze 30 cases of tuberculosis patients and 27 cases of pneumonia and compared the imaging results to evaluate the application value of MRI images in the identification of tuberculosis and pneumonia, aiming to provide a reference basis for clinical follow-up treatment and supply more effective inspection methods for the identification of tuberculosis and pneumonia.

## 2. Materials and Methods

### 2.1. Research Objects

30 tuberculosis patients and 27 pneumonia patients admitted to the hospital from March 2018 to March 2020 were selected as the research objects. All patients underwent MRI examinations with a noise reduction algorithm. There were 17 males and 40 females, and the age range of the patients was 18–73 years, with an average age of 37.54 ± 6.34 years. The diagnostic criteria were referred to the relevant diagnostic criteria in the *Diagnostic Standards and Management Practices of Tuberculosis* [13] and *Differential Diagnosis of Pneumonia* [14]. This study had been approved by the medical ethics committee of the hospital.

The inclusion criteria include patients who met the above diagnostic criteria, were not allergic to the relevant treatment and inspection drugs used in the treatment or examination in this study, and were aware of and signed the informed consent (their family members also signed that).

The exclusion criteria include patients who were combined with cognitive impairment, had poor compliance, were unable to cooperate with the researchers, recently received relevant drug treatment, and were accompanied with severe liver and kidney damage.

### 2.2. MRI Detection Method

Each patient was examined with an MRI diagnostic instrument, and the body was imaged with a phased array surface coil. The examinee took a supine position, put both hands on both sides of the body, placed the body coil in front of the chest wall, and wrapped the desired scanning range so that it covered the target area. The center of the front and back coils should be in a straight line. Then, an abdominal band was applied to fix with moderate strength. Without affecting the subject's breathing movement, it should ensure that the subject's body felt more comfortable to the utmost extent, and the abdominal band should try to be tightened. The patient should be instructed to carry out breath-holding training for no less than 18 seconds. All sequences adopted deep breathing and breath-hold scanning, including fast spin echo (FSE)/T1-weighted imaging (T1WI), FSE/T2WI sequence scanning, reverse recovery sequence scanning with short inversion time, and axial FSE/T2WI sequence scanning. The parameters were set as follows: the echo time during FSE/T1WI sequence scanning was 15–20 ms, and the repetition time was 470 ms; the echo time during FSE/T2WI sequence scanning was 130 ms, and the repetition time was 4,350 ms; the echo time during reverse recovery sequence scanning was 20 ms, and the repetition time was 5,635 ms; and the echo time during axis FSE/T2WI sequence scanning was 100 ms, and the repetition time was 4,475 ms. The scan slice spacing and slice thickness were both set to 5.2 mm, and some patients could undergo enhanced scanning after routine scanning. The examination range was referred to the location of the lesion on the positioning film to perform accurate lesion scanning. It took about 6–8 minutes to complete the routine scanning. The condition of the patient should be observed, and if there was any abnormality, stop immediately and give appropriate treatment.

### 2.3. Deep Convolutional Neural Network

The structure of DCNN is mainly improved from conventional CNN, and its structure is mainly composed of input layer, convolutional layer, activation function, another processing layer, and output layer.  Figure 1 shows the specific structure diagram.

The first part is the input layer. The main function of this layer is inputting data. The advantage of this layer is retaining the input image structure information.

The second part is the convolution layer, which uses the convolution kernel to process the input sample and extract the information of the sample. However, the change of convolution kernel is related to the depth of network structure, while the extraction of sample information is related to the depth of convolution layer position. The more features need to be extracted, the more distorted the display will be. The specific expressions are as follows.

Firstly, the noise characteristics should be extracted and counted, and the approximate model of noise is expressed as follows:

(1) $$\begin{array}{c} Ql=Ql-1◎xl+jl. \end{array}$$

In equation (1), *QL*-1 refers to the input sample information of layer 1, *◎* refers to the operation method of the convolution layer, *xl* refers to the number of layers of the convolution layer, JL refers to the input deviation, and *Ql* refers to the sample output information of layer 1 of the convolution layer.

The third part is the activation function, which is the most critical part of the DCNN structure and can introduce nonlinear operations into the whole model. Activation functions are other linear operations that add depth to the network and are the basis for the expression of the network. The propagation direction of the network is changed. When it shows reverse propagation, the gradient derivative obtained by it will be different from the change of activation function. In the DCNN structure, its specific operation expression is as follows:

(2) $$\begin{array}{c} Q=\frac{1}{\left(1+e-x\right)}, \end{array}$$

(3) $$\begin{array}{c} \text{tanh}\left(x\right)=\frac{\left(1-e-2x\right)}{\left(1+e-2x\right)}, \end{array}$$

(4) $$\begin{array}{c} Q=\left\{\begin{array}{c} x,\;x\geq 0\\ 0,\;x＜0 \end{array}\right). \end{array}$$

The fourth part is other processing layers, including the pooling layer and full connection layer. The main functions of the pooling layer are deleting redundant information, reducing feature mapping, thus further reducing the amount of computation, so that the basic information of the image remains in its original place. It can also assist the network model to prevent it from being too fit. At present, the main operation of the pooling layer is that the window regions do not overlap. Once pooled, it means that pooled regions at adjacent locations will be overlapped. Another phenomenon, known as pyramid pooling, enables convolution features of images at different scales to be in the same dimension. However, the fully connected layer generally belongs to the layer with the most parameters, because each node of this layer is connected with all nodes of the upper layer, which is fully connected.

The fifth part is the output layer, which adopts Softmax to directly convert and output the probability distribution values fully connected to each class.

In the whole training process, the loss of each round is calculated by the previous propagation and loss function, and then the backward propagation loss function continues to propagate. However, under the appropriate optimization, the loss can be effectively reduced, such as reducing the random gradient, reducing and updating parameters, and so on. In other words, the loss function has an important guiding significance for the whole network, and it has a great influence on the quality of the final learning result.

### 2.4. Image Processing

Using the above model, the obtained test images were automatically transmitted to the Siemens postprocessing workstation for noise reduction processing. An ADC image was synthesized from 3 MRI images with different *b* values, and the ADC value was directly measured.

The threshold of an image was divided into two parts (the foreground and the background), and the gray difference between the two was enlarged as much as possible. For an image *y* (*x*, *y*) with a size of *l* ∗ *n*, the initial threshold was set to *R*, the number of pixels in the pixel level *y*1 whose gray level was lower than the threshold was set to *n*_1_, and the number of pixels above the threshold was set to *n*_2_, which needed to be guaranteed *n*_1_ + *n*_2_ = *l* ∗ *n*, and the proportions of the two pixels had to satisfy *a* + *b* = 1:

(5) $$\begin{array}{c} a=\frac{n_{1}}{l*n},\\ b=\frac{n_{2}}{l*n}. \end{array}$$

The average gray level corresponding to the two parts was as follows:

(6) $$\begin{array}{c} a=\frac{\sum_{\left(k.d\right)\in n_{1}}n\left(k.d\right)}{n_{1}},\\ b=\frac{\sum_{\left(k.d\right)\in n_{1}}n\left(k.d\right)}{n_{2}}. \end{array}$$

In the previous equation, *n*(*k*.*d*) stood for the pixel value, from which the average gray value *z* of the entire image could be calculated:

(7) $$\begin{array}{c} z=z_{1}*a+z_{2}*b. \end{array}$$

The SNR of MRI images with different *b* values was compared, and the diagnostic efficacy of ADC values for solid lung lesions were analyzed to select the best *b* value. The observation and measurement of MRI images were carried out by 2 senior physicians in the imaging department. If there were different judgment results, it would be handed over to a third physician of the same level to assist in the solution.

### 2.5. Statistical Methods

The test data were processed using SPSS19.0 statistical software, and the measurement data were expressed as the mean ± standard deviation ($\bar{x}$ ± *s*). The comparison of the means between each group was performed by *t*-test. The count data were represented by percentage (%), and the *χ*^2^ test was adopted. In addition, *P* < 0.05 indicated that the difference was statistically substantial.

## 3. Results

### 3.1. MRI Imaging Results Based on Deep Learning Algorithm

Figure 2 is the MRI image of pneumonia, suggesting that the image before the noise reduction process was blurry, and the lung tissue and bronchus could not be clearly distinguished. The MRI image after the noise reduction algorithm was clearer, and the lung tissue was also clearer. The edges were regular, and the inflammatory signal was high.  Figure 3 shows the evaluation results of noise reduction. The signal-to-noise ratio (SNR) and carrier-to-noise ratio (CNR) of the MRI image after noise reduction were significantly better than those before processing (119.79 vs. 83.43, 12.59 vs. 7.21) (*P* < 0.05), indicating that the image noise reduction algorithm was effective.  Figure 4 displays the noise reduction process, meaning that the noise reduction algorithm could reduce the noise of the original image.

### 3.2. Comparison of the Baseline Data of All Patients

Table 1 indicates no statistical difference in the basic data between the tuberculosis group and the pneumonia group (*P* < 0.05).

### 3.3. MRI Imaging Results of the Patients

Figure 5 is an image of the combined sphere of the upper lobe of the lung. There were calcifications in the lesions, with satellite lesions around them and radial. ADC showed that the lesions were medium-signal, and some of the lesions were high-signal.  Figure 6 indicates the inflammatory lesions of the upper lobe of the lung. An elliptical soft tissue density shadow can be observed, with a striped shadow around it. The lesion was a high-signal shadow, while the ADC image at the corresponding level showed a low-signal shadow.  Table 2 shows that the accuracy of MRI based on deep learning algorithms in the diagnosis of tuberculosis and pneumonia (96.67% vs. 70%, 100% vs. 62.96%) was significantly improved (*P* < 0.05).

### 3.4. Comparison of SNR and CNR of MRI Images with Different *b* Values

Figure 7 shows the CNR and SNR of MRI images with different *b* values. When *b* = 0, the CNR and SNR were 10.44 and 14.29, respectively. When *b* = 500, the CNR and SNR were 6.23 and 8.95, respectively. When *b* = 800, CNR and SNR were 3.12 and 5.03, respectively. It revealed that as the b value increased, the CNR and SNR of MRI images showed a downward trend and the difference was statistically significant (*P* < 0.05).

## 4. Discussion

In recent years, the prevalence of lung diseases has gradually increased, tuberculosis has a tendency to reflame, and pneumonia has also become a highly infectious disease that needs to be closely prevented and controlled [15–17]. Studies have shown that tuberculosis is a highly infectious chronic lung disease [18, 19]. In clinical work, pulmonary tuberculosis is difficult to distinguish because of its similar clinical manifestations and pathological changes to pneumonia, especially in the early stages of the disease, it is often misdiagnosed, leading to delays in treatment [20]. In this study, the application value of deep learning MRI images in the identification and application of tuberculosis and pneumonia was explored, with a view to providing more examination methods for clinical identification and providing a supporting basis for its application effects.

Some researchers have adopted MRI in the diagnosis of tuberculosis and pneumonia, finding that invasive and proliferative pneumonia present the moderate signal in the examination sequence, there is a low signal in the cavity, and the signal is mostly uneven in tuberculoma [21, 22]. In this study, it was found that calcifications in the lesions were observed in the combined sphere imaging image of the upper lobe of the lung, and their surrounding was satellite lesions, which were radial. Then, ADC meant that the lesions had medium signals, and some lesions had high signals. An elliptical soft tissue density shadow could be observed in the upper pulmonary inflammatory lesions with a band shadow around it, the lesions were high-signal shadows, and the ADC images of the corresponding layers showed low-signal shadows. Therefore, it can be concluded that the signal of tuberculosis lesions and the signal of pneumonia consolidation were high in the sequence of MRI examinations, which was similar to the research findings of previous researchers [23].

In addition, the noise reduction algorithm in in-depth learning was used, in order to improve the accuracy of the MRI examination in this study. As a result, it was found that the MRI image processed by the noise reduction algorithm was clearer, with regular lung tissue edges and higher inflammation signals. The CNR and SNR were both high, indicating that the original image had a good imaging effect after noise reduction and correction. Arabi et al. [24] proposed that the DCNN method showed higher vulnerability to anatomical variation, and more outliers were observed in this method. Huo et al. [25] also proposed that MRI images processed by the DCNN method were more accurate in detecting splenic diseases. Moreover, it was concluded in this study that the accuracy of MRI based on deep learning algorithms in the diagnosis of tuberculosis and pneumonia (96.67% vs. 70%, 100% vs. 62.96%) was obviously improved (*P* < 0.05). The DCNN algorithms show good results in the processing of MRI images, and have high clinical application value, which is consistent with a large number of research results [26, 27].

## 5. Conclusion

Based on the deep learning noise reduction processing algorithm, the model was established and applied to MRI imaging results. In the process of identifying tuberculosis and pneumonia, the shadow of tuberculosis lesions under a specific sequence was higher than that of pneumonia. This reflected the importance of deep learning-based MRI images in the differential diagnosis of tuberculosis and pneumonia. The results of this study can provide a reference for clinical follow-up diagnosis and treatment. However, the shortcoming of this study was that it failed to make the display effect of MRI images more detailed, such as the difference in the display effects of the two diseases under each scan sequence of MRI, so it would be further studied in future work. To sum up, MRI images based on deep learning can effectively identify the pathological changes of tuberculosis and pneumonia, thereby providing a reference for clinical identification. It also indirectly suggested that the future development prospects of deep learning algorithms in the field of medical imaging were considerable, and they were worthy of clinical application and promotion.

## Figures and Tables

**Figure 1:** Schematic diagram of DCNN structure.

**Figure 2:** MRI imaging results based on the deep learning algorithm. (a) Before. (b) After.

**Figure 3:** Evaluation of noise reduction effect. Note. ^∗^ suggests the difference was statistically significant (*P* < 0.05).

**Figure 4:** Noise reduction processing results.

**Figure 5:** MRI results of tuberculosis.

**Figure 6:** MRI results of pneumonia.

**Figure 7:** The comparison results of SNR and CNR of MRI images with different *b* values. Note: ^∗^ and ^#^suggest that the change on CNR and SNR was statistically obvious with increase in *b* value, respectively (*P* < 0.05).

**Table 1:** Comparison of the baseline data of patients from the two groups.

Group	Tuberculosis group (*n* = 30)	Pneumonia group (*n* = 27)	*t* value or *χ*^2^ value	*P* value
Age (years old)	39.21 ± 1.12	39.06 ± 2.02	0.351	>0.05
Male (case (%))	8 (26.67)	9 (33.33)	0.302	>0.05
Female (case (%))	22 (73.33)	18 (66.67)	—	>0.05
Fever (case (%))	7 (23.33)	8 (29.63)	0.032	>0.05
Cough and expectoration (case (%))	5 (16.67)	4 (14.81)	0.000	>0.05
Hemoptysis (case (%))	8 (26.67)	6 (22.22)	0.002	>0.05

**Table 2:** MRI diagnosis accuracy rate based on the deep learning algorithm.

	Number of cases	MRI	MRI after optimization
Tuberculosis group	30	21 (70%)^*∗*^	29 (96.67%)^*∗*^
Pneumonia group	27	17 (62.96%)^*∗*^	27 (100%)^*∗*^

Note: ^*∗*^The difference was statistically significant (*P* < 0.05).

## Data Availability

The data used to support the findings of this study are available from the corresponding author upon request.
